# Fibrinogen Level Predicts Outcomes in Critically Ill Patients with Acute Exacerbation of Chronic Heart Failure

**DOI:** 10.1155/2021/6639393

**Published:** 2021-04-30

**Authors:** Zhongyuan Meng, Yaxin Zhao, Yan He

**Affiliations:** ^1^Guangxi Medical University, Nanning, Guangxi, China; ^2^The First Affiliated Hospital of Guangxi Medical University, Nanning, Guangxi, China

## Abstract

**Background:**

Heart failure (HF) is a common cardiovascular disease, which is related to systemic inflammation for decades. Fibrinogen (FIB) is a sign of thrombosis and inflammation, which is associated with the prognosis of many diseases. Nevertheless, the role of fibrinogen level in the prognosis of critically ill patients with acute exacerbation of chronic heart failure is unclear.

**Methods:**

The data are from the Medical Information Mart for Intensive Care III (MIMIC III) database, which is a freely accessible critical care database. The primary outcome in our study was 90-day mortality. The prognostic value of fibrinogen was analyzed with receiver operating characteristic (ROC) curve analysis, Kaplan-Meier curve, and Cox model.

**Results:**

A total of 554 patients were included. Patients were divided into two groups, low fibrinogen level (<284 mg/dl) and high fibrinogen level (≥284 mg/dl), through the cut-off value of the ROC curve. The area under the ROC curve of fibrinogen for predicting 90-day mortality was 0.65 (95% CI: 0.59–0.70). In the unadjusted Cox model, compared with the low fibrinogen level (<284 mg/dl), the 90-day mortality of the hazard ratio (HR) with 95% confidence intervals (CI) of the high fibrinogen level is 3.33 (95% CI 2.15-5.15). In different multivariable Cox models, compared with the low fibrinogen level (<284 mg/dl), the 90-day mortality of the hazard ratio of the high fibrinogen level is from 2.83 to 3.13. In subgroup analyses, significant interactions were observed only in age, chronic kidney disease (CKD), and APS III scores.

**Conclusion:**

Our data suggest that high fibrinogen levels (≥284 mg/dl) independently predict mortality in critically ill patients with acute exacerbation of chronic heart failure. Our findings need to be further validated by large prospective studies and longer follow-up time.

## 1. Introduction

Heart failure (HF) is a common cardiovascular disease, and the prevalence of heart failure has increased to 6.2 million in Americans over the age of 20 [1]. Heart failure is a disorder of the myocardial structure and function, which leads to restricted ventricular ejection or filling, impaired blood circulation throughout the body, and insufficient tissue and organ perfusion [2]. Heart failure has been seen to be related to systemic inflammation for decades [3, 4].

Fibrinogen (FIB) is produced by the liver and activated during the clotting process [5], which is a sign of thrombosis and inflammation [6]. In addition, fibrinogen is also related to the prognosis of many diseases, including coronary artery disease [7–9], diabetes [10, 11], and chronic kidney disease [12]. Fibrinogen levels were increased in patients with chronic cardiac insufficiency [13–15]. Nevertheless, most previous studies only analyzed how heart failure affects fibrinogen levels [16–18].

The influence of relative fibrinogen level on the prognosis of patients with acute exacerbation of chronic heart failure still lacks relevant research. Therefore, we intend to investigate the effect of the fibrinogen level on the prognosis of acute exacerbation of chronic heart failure. A better understanding of the relationship between fibrinogen level and acute exacerbation of chronic heart failure may help in risk stratification and assist in treatment to reduce mortality. The purpose of our study was to explore the effect of fibrinogen level on the prognosis of severe patients with acute exacerbation of chronic heart failure.

## 2. Methods

The data for all the studies are from the Medical Information Mart for Intensive Care III (MIMIC III) database, which is a freely accessible critical care database [19]. MIMIC III comprised about 60000 ICU admissions at the Beth Israel Deaconess Medical Center in Boston. All subjects' names were replaced by subject_id, which fully protects the patient's privacy. The information recorded in the database includes demographic characteristics, diagnosis, laboratory examination data, microbial culture data, imaging data, nursing records, treatment measures, and fluid balance. After completing the National Institutes of Health web-based training course, we are eligible to access the database. Data were extracted by author Meng who has completed an online training course at the National Institutes of Health (Zhongyuan Meng, certification number: 9071533).

### 2.1. Subjects Selection

We selected all patients in the database with the first ICU admission. The inclusion criteria were the following: (1) the patients were older than 18 years old, (2) the patients stayed in ICU more than 24 hours, (3) the patients had acute exacerbation of chronic heart failure, and (4) the patients had data on the fibrinogen.

### 2.2. Data Extraction

Data extracted from the MIMIC III database includes gender, age, ethnicity, BMI, mean blood pressure, sequential organ failure assessment (SOFA) score, Acute Physiology Score III (APS III score), Systemic Inflammatory Response Syndrome (SIRS score), Simplified Acute Physiology Score II (SAPS II score), vasopressor use, ventilator use, date of hospital admission and discharge, date of ICU admission and discharge, and date of birth and death. Comorbidities included atrial fibrillation (Af), high blood pressure (HBP), diabetes mellitus (DM), chronic kidney disease (CKD), acute kidney injury (AKI), respiratory failure, and acute myocardial infarction (AMI). Laboratory examination includes hemoglobin (Hb), platelet (PLT) count, white blood cell (WBC) count, fibrinogen, serum creatine (Scr), NT-proBNP, and serum glucose. All data were the results of the patient's initial examination after hospital admission. As there are too many missing records of NT-proBNP, we converted it into a dummy variable in the model. The primary outcome in our study was 90-day mortality, defined as death occurring within 90 days after admission. In addition, we made a preliminary assessment of 28-day mortality and ICU length of stay (LOS).

### 2.3. Statistical Analyses

The measurement data consistent with normal distribution were expressed as mean ± standard deviation, and the comparison between groups was performed by the *t*-test. Nonnormally distributed data were represented by median and interquartile difference (IQR), and the Wilcoxon rank sum test was used for comparison between groups. The categorical variables are presented by frequency and used by the chi-square test. The receiver operating characteristic (ROC) curve analysis, Kaplan-Meier curve, and Cox proportional hazards models were performed to determine the association between fibrinogen and 90-day mortality. ROC results showed that the cut-off value of fibrinogen predicting 90-day mortality was 284 mg/dl. Thus, the study population was divided into two groups, namely, low fibrinogen group (<284 mg/dl group) and high fibrinogen group (≥284 mg/dl group) according to fibrinogen. The low fibrinogen level was selected as the reference group. To control the influence of confounders, we choose multivariable analysis to adjust. Multicollinearity was tested by a variance inflation factor (VIF). VIF ≥ 5 indicated the existence of multicollinearity. Model 1 was adjusted for only fibrinogen, PLT, NT-proBNP, vasopressor use, and ventilator use. Model 2 = model 1+HBP, Af, respiratory failure, chronic kidney disease, and STEMI. Due to the multicollinearity in each severe disease score, only one score is added to each model for correction. Model 3 = model 2+SIRS scores (VIF 4.24). Model 4 = model 2+APS III scores (VIF 3.94). Model 5 = model 2+SAPS II scores (VIF 4.22). Stata16 MP was used for statistical analysis of all data; a two-side *P* < 0.05 was considered statistically significant.

## 3. Result

554 patients met the inclusion criteria. The flowchart of patient selection is shown in Figure 1.  Table 1 lists the basic characteristics of all patients by the low fibrinogen group (<284 mg/dl group) and high fibrinogen group (≥284 mg/dl group). There were 225 patients in the low fibrinogen group and 329 patients in the high fibrinogen group. The high fibrinogen group tended to have high PLT count, high Scr, HBP, CKD, STEMI, vasopressor use, ventilator use, high APS III, SAPS II, and SIRS scores.  Figure 2 shows the ROC curves of fibrinogen and different severity scores. In all ROC curves, the area of AUC is less than 0.7. However, after combining fibrinogen and SAPS II, the AUC of the joint prediction model reaches 0.73 (95% CI 0.69-0.78), which is higher than that of fibrinogen and other disease severity scores alone.

Figure 3 shows the Kaplan-Meier curve for patients in the low and high fibrinogen groups. A higher fibrinogen was significantly associated with risk of 90-day mortality (*P* < 0.0001 by the logrank test). In Table 2, we use the Cox model to analyze the association between fibrinogen and 90-day mortality. In the unadjusted Cox model, compared with the low fibrinogen group, the 90-day mortality of HR (95% CI) of the high fibrinogen group is 3.33 (95% CI, 2.15-5.15). In the extended multiple COX model, high fibrinogen levels were significantly associated with increased 90-day mortality, in model 1 (HR 3.35, 95% CI 1.95-5.76), model 2 (HR 3.11, 95% CI 1.81-5.36), model 3 (HR 3.13, 95% CI 1.82-5.40), model 4 (HR 2.83, 95% CI 1.63-4.90), and model 5 (HR 2.85, 95% CI 1.65-4.92).

### 3.1. Subgroup Analysis

Subgroup analysis was used to assess association between fibrinogen and 90-day mortality in different groups (Table 3). Significant interactions were observed in age, CKD, and APS III scores. For patients ≥ 65 years old, the risk of 90-day mortality was significantly higher in the high fibrinogen group (HR 4.16, 95% CI 2.51-6.88), whereas we did not find this relationship in patients < 65 years old (HR 1.29, 95% CI 0.50-3.28). In patients without CKD, the risk of 90-day mortality was significantly higher in the high fibrinogen group (HR 9.87, 95% 3.91-24.8). Similarly, in the APS III scores < 48 group, the risk of 90-day mortality was significantly higher in the high fibrinogen group (HR 7.69, 95% 2.69-21.9).

## 4. Discussion

At present, there are few studies to report the effect of fibrinogen on the prognosis of acute exacerbation of chronic heart failure. In the current study, we explored the connection between fibrinogen levels and the prognosis of patients with acute exacerbation of chronic heart failure. In our study, we found that fibrinogen levels ≥ 284 mg/dl had a significant correlation with mortality. Compared to the prediction accuracy of fibrinogen with different severe disease scores, we observed that only SAPS II and APS III had a slightly higher predictive accuracy than fibrinogen. However, the acquisition of SAPS II and APS III requires measurement of multiple data, including not only general vital signs but also blood gas analysis results, etc. Therefore, these difficulties bring certain challenges to clinical use. On the contrary, fibrinogen is an easy-to-measure indicator, which is convenient for clinical use. Of course, we can also significantly improve the prediction accuracy when we combine fibrinogen and disease severity scores.

In contrast to our findings, Chin et al. [20] studied 120 outpatients with chronic stable heart failure and found that there was no significant correlation between fibrinogen levels and all-cause mortality. There are several factors that may contribute to the inconsistencies in the results. We studied critically ill patients with acute episodes of chronic heart failure, while Chin et al. studied patients with chronic stable heart failure. Outcomes between different cohorts may also vary greatly. Our cohort study revealed that patients with acute episodes of chronic heart failure at a higher level of fibrinogen (threshold value > 284 mg/dl) had a higher risk of 90-day mortality compared to patients with a lower level. In our study, after adjusting the related covariates, high fibrinogen levels still showed a strong correlation with 90-day mortality (HR from 2.83 to 3.13, *P* < 0.0001).

There is increasing evidence that fibrinogen is a poor prognostic predictor of cardiovascular disease. Fibrinogen may increase cardiovascular risk through platelet aggregation, plasma viscosity, and fibrin formation [21]. Stec et al. [22] measured fibrinogen levels in 2,632 subjects using a newly developed immunoprecipitation test; they suggest that fibrinogen is associated with traditional cardiovascular risk factors. A study by Kotbi et al. [23] has also shown that fibrinogen is related to the severity of coronary artery disease and cardiovascular risk in Moroccan patients. A large meta-analysis found a moderately strong correlation between plasma fibrinogen levels and coronary heart disease risk [24]. In addition, Song et al. [6] suggested that fibrinogen was an independent predictor of reinfarction after PCI in NSTE-ACS patients. After adjusting for variates, FIB level also is associated with a higher rate of death/nonfatal reinfarction (HR = 1.498, 95% CI: 1.030-2.181, *P* = 0.035). Although these studies are different, most of the conclusions reached are very similar to our research; that is, fibrinogen is closely related to the prognosis of cardiovascular disease.

We studied the possibility of the relationship between fibrinogen and mortality in patients with acute exacerbation of chronic heart failure. Fibrinogen is easy to obtain and convenient for clinical use. Admission fibrinogen measurement may be used to stratify the prognosis risk of acute exacerbation of chronic heart failure and provide a reference for later treatment. To our knowledge, this seems to be the first study to evaluate the relationship between fibrinogen and the prognosis of acute exacerbations of chronic cardiac function, and this may be helpful for clinical practice.

### 4.1. Study Limitation

Our study had several limitations. Although we found that high fibrinogen is independently associated with adverse outcomes, our study is still a single-center retrospective study. We only collected the data of the patient on admission. The relationship between the dynamic changes of fibrinogen and patients with acute exacerbation of chronic heart failure cannot be analyzed.

## 5. Conclusion

Our data suggest that high fibrinogen levels (≥284 mg/dl) independently predict mortality in critically ill patients with acute exacerbation of chronic heart failure. Our findings need to be further validated by large prospective studies and longer follow-up time.

## Figures and Tables

**Figure 1:** The flowchart of patient selection.

**Figure 2:** Receiver operating characteristic curves of fibrinogen and severity scores for predicting 90-day mortality.

**Figure 3:** Kaplan-Meier curves for 90-day mortality.

**Table 1:** Summary of patient characteristics.

	Total (*n* = 554)	Fibrinogen level < 284 mg/dl (*n* = 225)	Fibrinogen level ≥ 284 mg/dl (*n* = 329)
Age (years)	72.2 ± 13.7	71.4 ± 12.8	72.7 ± 14.2
BMI (kg/m^2^)	28.7 ± 6.4	28.1 ± 5.8	29.1 ± 6.7
Gender (male), *n* (%)	319 (57.6)	124 (55.1)	195 (59.3)
*Ethnicity,n* (%)			
White	426 (76.9)	174 (77.3)	252 (76.6)
Black	33 (6.0)	12 (5.3)	21 (6.4)
Other	95 (17.1)	39 (17.3)	56 (17.0)
Mean BP (mmHg)	73.4 ± 9.1	72.7 ± 7.7	73.8 ± 10.0
*Laboratory outcomes*			
WBC count (10^9^/l)	13.1 ± 6.6	13.3 ± 5.9	12.9 ± 7.1
Hb (mg/dl)	10.0 ± 2.2	9.8 ± 2.5	10.2 ± 2.0
Scr (mg/dl)	1.5 ± 1.1	1.2 ± 0.7	1.7 ± 1.3
NT-ProBNP, *n* (%)	70 (12.6)	12 (5.3)	58 (17.6)
Platelet count (10^9^/l)	195.9 ± 100.8	164.7 ± 74.1	217.2 ± 110.8
Glucose (mg/dl)	152.8 ± 66.3	150.1 ± 63.7	154.7 ± 68.1
Fibrinogen (mg/dl)	371.1 ± 198.3	200.4 ± 53.1	487.8 ± 175.3
*Comorbidities*, *n* (%)			
Respiratory failure, *n* (%)	185 (33.4)	46 (20.4)	139 (42.2)
HBP, *n* (%)	265 (47.8)	121 (53.8)	144 (43.8)
DM, *n* (%)	224 (40.4)	84 (37.3)	140 (42.6)
Af, *n* (%)	291 (52.5)	123 (54.7)	168 (51.1)
AKI, *n* (%)	512 (92.4)	210 (93.3)	302 (91.8)
CKD, *n* (%)	273 (49.3)	89 (39.6)	184 (55.9)
NSTEMI, *n* (%)	131 (13.6)	47 (20.9)	84 (25.5)
STEMI, *n* (%)	32 (5.8)	7 (3.1)	25 (7.6)
Vasopressor use, *n* (%)	403 (72.7)	177 (78.7)	226 (68.7)
Ventilator use, *n* (%)	427 (77.1)	192 (85.3)	235 (71.4)
CRRT	41 (7.4)	11 (4.9)	30 (9.1)
*Disease scores*			
SOFA scores	6 (4-9)	4 (7-9)	6 (4-8)
APS III scores	48 (35-63)	42 (31-58)	52 (40-67)
SAPS II scores	42 (35-52)	40 (34-51)	44 (35-53)
SIRS scores	3 (2-4)	3 (2-3)	3 (3-4)
*Outcome*			
ICU LOS (days)	4.9 (2.7-8.6)	3.3 (2.5-6.1)	6.1 (3.2-10.2)
28-day mortality, *n* (%)	82 (14.8)	15 (6.7)	67 (20.4)
90-day mortality, *n* (%)	133 (24.0)	25 (11.1)	108 (32.8)

**Table 2:** Association between fibrinogen and 90-day mortality.

	Fibrinogen level (mg/dl)	Hazard ratio	95% CI	*P* value
Crude	<284	Ref		<0.0001
	≥284	3.33	2.15-5.15	
Model 1	<284	Ref		<0.0001
	≥284	3.35	1.95-5.76	
Model 2	<284	Ref		<0.0001
	≥284	3.11	1.81-5.36	
Model 3	<284	Ref		<0.0001
	≥284	3.13	1.82-5.40	
Model 4	<284	Ref		<0.0001
	≥284	2.83	1.63-4.90	
Model 5	<284	Ref		<0.0001
	≥284	2.85	1.65-4.92	

Adjusted covariates: model 1 = fibrinogen, PLT, NT-proBNP, vasopressor use, and ventilator use; model 2 = model 1+HBP, Af, respiratory failure, CKD, and STEMI; model 3 = model 2+SIRS scores (VIF 4.24); model 4 = model 2+APS III scores (VIF 3.94); model 5 = model 2+SAPS II scores (VIF 4.22).

**Table 3:** Subgroup analysis of the associations between fibrinogen and 90-day mortality.

Subgroup	*N*	HR (95% CI) <284 mg/dl	HR (95% CI) ≥284 mg/dl	*P* for interaction
Gender				0.198
Male	235	Ref	4.70 (2.30-9.57)	
Female	319		2.60 (1.50-4.53)	
Age				0.030
<65	149	Ref	1.29 (0.50-3.28)	
≥65	405		4.16 (2.51-6.88)	
HBP				0.066
Yes	265	Ref	5.42 (2.55-11.51)	
No	289		2.29 (1.34-3.91)	
DM				0.116
Yes	224	Ref	2.21 (1.16-4.21)	
No	330		4.46 (2.46-8.09)	
Af				0.388
Yes	291	Ref	3.97 (2.23-7.09)	
No	263		2.68 (1.38-5.20)	
Respiratory failure				0.346
Yes	185	Ref	2.16 (1.14-4.11)	
No	369		3.28 (1.80-5.97)	
CKD				0.001
Yes	273	Ref	1.61 (0.97-2.67)	
No	281		9.87 (3.91-24.8)	
AKI				
Yes	512	Ref	3.36 (2.17-5.20)	
No	42		NA	
NSTEMI				0.992
Yes	131	Ref	3.31 (1.27-8.63)	
No	423		3.35 (2.05-5.46)	
STEMI				0.161
Yes	32	Ref	1.12 (0.23-5.30)	
No	522		3.53 (2.24-5.56)	
Vasopressor use				0.304
Yes	403	Ref	3.81 (2.31-6.30)	
No	151		2.29 (0.94-5.54)	
Ventilator use				0.085
Yes	427	Ref	4.00 (2.43-6.60)	
No	127		1.63 (0.67-3.94)	
CRRT use				0.111
Yes	41	Ref	1.59 (0.64-3.96)	
No	513		3.63 (2.21-5.98)	
SOFA scores				0.293
<6	234	Ref	4.95 (2.11-11.60)	
≥6	320		2.86 (1.71-4.79)	
APS III scores				0.023
<48	271	Ref	7.69 (2.69-21.9)	
≥48	283		1.96 (1.21-3.17)	
SAPS II scores				0.966
<42	271	Ref	3.16 (1.44-6.94)	
≥42	283		3.05 (1.80-5.15)	
SIRS scores				0.845
<3	150	Ref	3.57 (1.45-8.78)	
≥3	404		3.20 (1.94-5.26)	

## Data Availability

The data used in the study is available at https://mimic.physionet.org/.

## Abbreviation

HF: Heart failure
BMI: Body mass index
Af: Atrial fibrillation
AMI: Acute myocardial infarction
Scr: Serum creatine
LOS: Length of stay
HR: Hazard ratio
CI: 95% confidence intervals
SOFA: Sequential organ failure assessment
APS III: Acute Physiology Score III
SIRS: Systemic Inflammatory Response Syndrome
SAPS II: Simplified Acute Physiology Score II
DM: Diabetes mellitus
CKD: Chronic kidney disease
AKI: Acute kidney injury
Hb: Hemoglobin
PLT: Platelets
WBC: White blood cells
FIB: Fibrinogen.
